# Evaluation of Financial Subsidy for Agriculture Based on Combined Algorithm

**DOI:** 10.1155/2022/6587460

**Published:** 2022-06-01

**Authors:** Kexin Chen, Zhenyu Wang

**Affiliations:** ^1^College of Economics and Management, Shenyang Agricultural University, Shenyang 110866, Liaoning, China; ^2^Business School, Shenyang University, Shenyang 110044, Liaoning, China; ^3^School of Economics, Liaoning University, Shenyang 110036, Liaoning, China

## Abstract

The stable development of agriculture is related to the national economy, and the fragility and foundation of agricultural production determine the inherent requirements of the government for financial support of agriculture. Based on China's policy of agricultural subsidy, in this study, the basic characteristics and classification methods of agricultural subsidies are analyzed, and an evaluation model of agricultural subsidies is established based on a combined algorithm, where the attributes of agricultural subsidies are screened by analytic hierarchy process, and the evaluation process of agricultural subsidies is constructed by data envelopment approach. Moreover, the development level of regional financial subsidies for agriculture is measured by relative efficiency value, and the implementation direction of financial subsidies is evaluated, to enhance the administrative benefits of government finance and deepen the supply-side reform of agricultural financial subsidies, which promote the sustainable development of agricultural insurance and agricultural production.

## 1. Introduction

Agriculture is the foundation of human existence, which provides necessary conditions for all production activities, and is the foundation of social stability and economic development. However, agricultural production is restricted by the natural environment with inherent weakness, low efficiency, and high risk. At the same time, with the marketization of China's socialist economy, the problem of “agriculture, rural areas, and rural residents” has become increasingly prominent [1–3]. Therefore, in recent years, the Central Committee of the Communist Party of China has issued a series of policies to strengthen agriculture and benefit farmers, where the financial support and protection for agriculture, rural areas, and rural residents have been continuously enhanced. A subsidy is the way that the government provides transferred payment to the production, circulation, and trade of agricultural products through administrative means [4, 5]. It helps to support and protect the agricultural field, which plays a very important role in promoting agricultural development, healthy operation of national economy, and protecting farmers' interests, and occupies an important position in the economic policies in the world.

However, there are many outstanding problems of supply-side structural contradictions in China's agricultural development at present. Although the total amount of grain is increasing continuously, due to the change in social demand, the imbalance of supply, and demand structure of agricultural products, the costs of agricultural production has been rapidly increased, and the comparative benefits and internal motivation of agricultural development are obviously weakened [6–8]. For a long time, China's cultivated land resources have been relatively short. Under the condition of overexploitation of cultivated land and serious pollution, the pressure on agricultural resources and environment has become greater. In addition, some policies of agricultural subsidy are biased in pertinence due to imperfect guiding mechanism, which leads to the continuous weakening of agricultural subsidies.

The performance evaluation of agricultural subsidies refers to the use of a method or model to measure the efficiency of agricultural financial subsidies and to measure the achievement of government performance in the process of agricultural financial subsidies or the governance efficiency of government in the process of agricultural development participation [9, 10]. Through the results of performance evaluation, the shortcomings can be found in the process of government administration, which provides guidance for the improvement and stable implementation of the follow-up agricultural financial subsidies.

## 2. Basis of Agricultural Subsidies

Agricultural subsidies are part of financial subsidies, by implementing specific financial support for some specific projects, and according to certain subsidy basis and standards, the supply and demand structure of agricultural products and agricultural means of production is changed, thus generating the income effect and substitution effect, which is a kind of transfer expenditure of the government with guiding function.

### 2.1. Basic Characteristics of Agricultural Subsidies

From the connotation of the abovementioned agricultural subsidy policy, it can be known that the characteristics of agricultural subsidy policy mainly include the following points [11–14]:

1. The main body of agricultural subsidy policy is the government. No matter what kind of agricultural subsidies are adopted, the subsidy funds will ultimately come from fiscal revenue.
2. Agricultural subsidy belongs to the government's transfer expenditure; that is, it is a unilateral and unpaid transfer of funds given by the government to agricultural producers, consumers, or operators. Agricultural producers, consumers, or operators who get agricultural subsidies will inevitably get certain benefits that are not equivalent. A subsidy is a kind of pure benefit increase or cost decrease, so agricultural subsidy must be a behavior of transfer payment.
3. The policy objectives of agricultural subsidies are often diversified and phased. There are three main objectives of agricultural subsidy policy: ensuring food security; raising farmers' income level; and realizing the sustainable development of agriculture and rural economy, which will be adjusted correspondingly with the changes in economic development level, industrial structure, and other related economic variables.
4. Agricultural subsidies are diversified and flexible. The diversified characteristics of agricultural subsidy policy inevitably require that agricultural subsidy methods have both diversity and flexibility.

### 2.2. Classification of Agricultural Subsidies

As shown in Figure 1, according to different classification standards, agricultural subsidy policies can be classified in many different ways. In the light of different links of agricultural production, subsidy policies can be divided into productive subsidies, circulation subsidies, and income subsidies, while according to different payment methods, agricultural subsidy policies can be divided into direct subsidy and indirect subsidies [15–17]. Meanwhile, according to different subsidy objects, it can be divided into producer subsidy, consumer subsidy, and operator subsidy.

According to the functional mechanism of agricultural subsidies, this study divides them into four types: income-based agricultural subsidies, cost-based agricultural subsidies, technology-based agricultural subsidies, and price-based agricultural subsidies, as shown in Figure 2.

#### 2.2.1. Income-Based Agricultural Subsidies

It refers to the agricultural subsidy policy that directly subsidizes farmers to increase their income, thus affecting the total expenditure of farmers' agricultural budget. Hook grain direct subsidies and Hook comprehensive agricultural resources subsidies belong to income-based agricultural subsidies, while unhook grain direct subsidy generally takes the taxable farmland or taxable regular production as the basis of grain direct subsidy, where whether farmers actually plant or not, there is subsidy when there is contracted land, which is a kind of inclusive subsidy and belongs to income-based agricultural subsidy policy. The way and mechanism of unhook agricultural comprehensive subsidies are similar to those of unhook grain direct subsidies, so unhook agricultural comprehensive subsidies also belong to income agricultural subsidies.

#### 2.2.2. Cost-Based Agricultural Subsidies

By reducing the cost of grain production, it can mobilize farmers' enthusiasm for growing grain, which promotes the increase in grain production and increases farmers' income level. Unhook direct grain subsidies and unhook comprehensive agricultural subsidies are cost-based agricultural subsidies. Hook grain direct subsidy means that the grain direct subsidy is linked to the current agricultural production and planting situation; that is, linked grain direct subsidy is subsidized according to the actual grain planting area of farmers, and the amount of direct grain subsidy is linked to the planting area. Hook grain direct subsidy can reduce the cost of grain production, mobilize farmers' enthusiasm for growing grain, and thus promote the increase in grain production and farmers' income, so it is a cost-based agricultural subsidy policy. The same argument, hook comprehensive agricultural subsidies also belong to the cost-based agricultural subsidy.

#### 2.2.3. Technology-Based Agricultural Subsidies

It refers to the policy that advances the agricultural production mode through new products and technologies, thus improving the production efficiency of agricultural products. Improved varieties' subsidy, farm machinery purchase subsidies, etc., are technology-based agricultural subsidies. Improved varieties' subsidy is a subsidy given by the government to farmers who use high-quality seed, which guides farmers to adopt new varieties and technologies and improves the output and quality of agricultural products, while farm machinery purchase subsidy is a subsidy given by the government to farmers who purchase farm machinery within the scope specified in the catalogue, which encourages and supports farmers to use advanced and applicable farm machinery, improves the mechanization process, and thus increases the output of agricultural products. Therefore, it belongs to the technology-based agricultural subsidies.

#### 2.2.4. Price-Based Agricultural Subsidies

It refers to the policy that promotes the development of grain production, protects farmers' enthusiasm for growing grain, and guarantees farmers' income from growing grain by stabilizing or influencing the prices of agricultural products, where the minimum purchase price, temporary purchasing and storage price, etc., are price-based agricultural subsidies.

## 3. Evaluation Model of Agricultural Subsidy Based on Combined Algorithm

### 3.1. Screen of Agricultural Subsidy Attribute Based on AHP

Analytic hierarchy process (AHP) is a process of modeling and quantifying the decision-making thinking process of decision-makers on complex systems, which is a hierarchical weight decision analysis method combining qualitative and quantitative analysis, where the decision-maker points out the standard weight of each decision scheme and calculates the ranking of the alternatives using the weight of each decision scheme [18]. According to the classification of subsidy mentioned above, the analytic hierarchy process adopted in this study is divided into the steps as shown in Figure 3.

#### 3.1.1. Establish a Hierarchical Structure Model

The targets, factors, and objects are divided into target level, criterion level, and scheme level according to their relationships, and the hierarchical structure is shown in Figure 4.

The decision-makers point out the weight of each scheme and then adopt the weight to calculate the ranking of the advantages and disadvantages of each alternative scheme. When there are many factors at a certain level, the layer can be further divided into sublayer orders of the next order [19].

#### 3.1.2. Construct a Judgment Matrix

The judgment matrix compares each other between pairwise, which is to reduce as little as possible the difficulty of comparing various factors due to different nature, thus improving the accuracy of the decision-making model. Assume that the elements of the judgment matrix are *a*_*ij*_, which is generally given by the Saaty 1–9 scale method, where *i* and *j* are horizontal and vertical coordinates, respectively. When using the numerical ratio with practical significance, the construction of the judgment matrix can express the importance degree between pairwise.

#### 3.1.3. Hierarchical Single Sorting and Its Consistency Test

The judgment matrix established in the second step is solved. The formula for characteristic root is as follows: $\bar{\text{A}}\text{W}=\lambda_{\max}W$ The eigenvector of *W* is obtained, the hierarchical single sort is solved, and the consistency of hierarchical single sort is checked. Here, you can define the consistency index formula (Cl). The formula is as follows, where *n* is the order of the judgment matrix.

When solving the characteristic root of judgment matrix $\bar{A}$, which has been established in the second step, the eigenvector *W* can be obtained in the formula $\bar{\text{A}}\text{W}=\lambda_{\max}W$. Then, the consistency test of a single order of levels is implemented; here, the consistency index formula Cl is defined as follows, where *n* is the order of the judgment matrix:

(1) $$\begin{array}{c} \text{CI}=\frac{\lambda_{\max}-n}{n-1}. \end{array}$$

The consistency ratio (CR) is defined, and its calculation formula is as follows:

(2) $$\begin{array}{c} \text{CR}=\frac{\text{Cl}}{\text{RI}}. \end{array}$$

When the consistency ratio CR < 0.1, it is considered that the degree of inconsistency of hierarchical single sorting is within the allowable range, and the result has satisfactory consistency; otherwise, the scoring matrix should be reconstructed [20].

#### 3.1.4. Hierarchical Total Sorting and Consistency Test

In this study, it is assumed that the upper level *A* contains *m* factors, which are *A*_1_, *A*_2_,…, *A*_*m*_, respectively, and then, the total sorting weights of these elements are *a*_1_, *a*_2_,…, *a*_*m*_, respectively. In addition, it is assumed that the next level B of the elements in the upper level contains *n* factors, which are *B*_1_, *B*_2_,…, *B*_*n*_, and then the single sorting weights of these elements for factor *A*_*j*_, including *b*_1*j*_, *b*_2*j*_,…, *b*_*nj*_ (if *B*_*k*_ and *A*_*j*_ are not related, *b*_*kj*_=0).

If in hierarchy *B* the consistency index of the hierarchical single ordering of element *A*_*j*_ of some factors is CI_*j*_, then the average random consistency index corresponding to these elements is RI_*j*_, and the calculation formula of the random consistency ratio of the total ordering of element *B* is shown as follows:

(3) $$\begin{array}{c} \text{CR}=\frac{\sum_{j=1}^{m}a_{j}{\text{CI}}_{j}}{\sum_{j=1}^{m}a_{j}{\text{RI}}_{j}}. \end{array}$$

### 3.2. Process of Agricultural Subsidy Evaluation Based on Data Envelopment Analysis

As shown in Figure 5, the experimental process of data envelopment method can be divided into four modules [21, 22].

#### 3.2.1. Define Data Variables

It consists of two parts: “determine the evaluation target” and “select the decision-making unit.” The evaluation target of this study is to realize performance evaluation of the government's agricultural financial subsidy policy, whose experimental process mainly refers to DEA, where the input and output of different subsidy categories are selected as decision-making units, including income subsidies, cost subsidies, technology subsidies, and price subsidies.

#### 3.2.2. Determine the Objective Function

It is mainly to establish input and output target system, which is mainly based on a decision-making unit of the module, where the input target and output target systems are based on the selection of AHP indicators, and the indicators in data envelopment method are established as shown in Figure 6.

The determined index system takes the per capita net income of rural residents, the proportion of agricultural employees, the average household population, the per capita common cultivated land area, the amount of chemical fertilizer used per acre, and the effective irrigated cultivated land area as the input indexes of decision-making unit in DEA and takes the agricultural development status, cultivated land endowment, rural labor force, and production factors as the output indexes of DEA decision-making unit.

#### 3.2.3. Choose DEA Model

CCR model is selected as the performance evaluation model of agricultural insurance financial subsidy. CCR model assumes that the production technology of the decision-making unit is constant to scale return and determines whether the decision-making unit is DEA effective by constructing production front.

#### 3.2.4. Establish Constraints

This module is the regulating variable in the whole performance evaluation process of agricultural financial subsidies, which controls whether the evaluation results are recognized by evaluators or relevant agricultural participants. Model participants can set constraint thresholds according to the existing experience of agricultural subsidies policies. If the evaluation results are accepted, the effectiveness of the DEA evaluation model is recognized and the model evaluation can be implemented. Otherwise, Step 3 is returned, the evaluation model is replaced or the AHP algorithm is adjusted to alter the evaluation index system, and then Step 4 is restarted.

### 3.3. Evaluation Model of Agricultural Financial Subsidies Based on Combination Algorithm

As shown in Figure 7, the evaluation model of agricultural financial subsidies proposed in this study is mainly divided into two modules: AHP module and DEA module, in which the main function of AHP module is to determine the evaluation index of DEA module; and DEA module establishes the evaluation target system according to the results of AHP, thus determining each decision-making unit and then evaluating agricultural financial subsidies.

The third-order hierarchical model of evaluation index is constructed as shown in Figure 8, in which the first-level index is the evaluation index system of agricultural financial subsidy policy that is also the target level of this evaluation index, the second-level index system includes scale index, efficiency index, influence index, and sustainability index, and the third-level index is the basic index related to the evaluation of agricultural financial subsidy.

The hierarchical total sorting of all judgment matrices is carried out by the index weight values under the single sorting of each level through the consistency test, and the results of the hierarchy total sorting are checked for consistency, as shown in Table 1.

## 4. Results and Discussion

The decision-making units in this study included income subsidies, cost subsidies, technology subsidies, and price subsidies. According to the results in Table 1, in the ranking of three-level indicators, four indicators with a comprehensive score greater than 0.1 are selected: the amount of financial subsidies, regional per capita income, economic development density, and economic development depth, and the amount of financial subsidies is taken as the input index of DEA decision-making unit, while regional per capita income, economic development density, and economic development depth are taken as the output indicators of DEA decision-making unit. Therefore, the settings of each unit are shown in Table 2.

Relative efficiency is the performance of agricultural insurance financial subsidies related to input index and output index, which can be used as a significant evaluation index to measure the effect of agricultural insurance fiscal subsidies in a certain region. According to the relevant data on agricultural fiscal subsidies provided by the Department of Finance (2015–2021), the input weight vector and output weight vector are calculated and the relative efficiency is calculated according to the evaluation input index and decision unit setting. The results are shown in Table 3.

The above results show that the relative efficiency of agricultural financial subsidies in this region is relatively high, and its comprehensive efficiency exceeds 0.9. Among them, the comprehensive efficiency of income subsidies is the best, which is 0.9832, while that of technological progress subsidies is lower, which is 0.9023. From the relative efficiency index of financial subsidies, the progress of related technologies has effectively promoted the improvement of agricultural productivity. In addition, according to the result of input-output efficiency value, the region still needs to strengthen the innovation of agricultural financial subsidy system, adjust the allocation structure of financial subsidy funds, and improve the allocation management of financial subsidy funds to make up for the lack of scale efficiency. Moreover, with the implementation of the financial subsidy policy, the stable development of subsidies has better compensated for the economic losses in the process of agricultural production and ensured the healthy production of agriculture.

It can be seen that China is in the new normal period of economy, the market puts forward higher requirements for the quality and safety of agricultural products, and the contradiction between market constraints and resources and environment faced by the development of agricultural industry is prominent, so it is urgent to promote the structural reform of agricultural supply side. Meanwhile, we should strengthen the implementation of technical subsidy policies and advance the rapid development of key agricultural technologies.

## 5. Conclusion

The evaluation of agricultural subsidies can improve China's agricultural management and promote the agricultural production with sustainable, healthy, and stable development. Therefore, this study establishes an evaluation model of agricultural subsidies based on a combined algorithm and measures the development level of regional agricultural financial subsidies with relative efficiency value. The evaluation result shows that in the hierarchical total sorting, the comprehensive score of financial subsidy amount, regional per capita income, economic development density, and economic development depth is greater than 0.1, which can be used as the decision-making unit of this model. The relative efficiency of agricultural financial subsidies in this region is relatively high, and its comprehensive efficiency exceeds 0.9. Among them, the comprehensive efficiency of income subsidies is the best, which is 0.9832, while the efficiency of technology-based subsidies is lower, which is 0.9023. The government should adjust the allocation structure of financial subsidy funds and strengthen the implementation of technical subsidy policies, to ensure the healthy production of agriculture.

## Figures and Tables

**Figure 1:** Classification of agricultural subsidies.

**Figure 2:** Classification of agricultural subsidies based on mechanism of action.

**Figure 3:** Steps of AHP based on classification of agricultural subsidies.

**Figure 4:** AHP hierarchy.

**Figure 5:** Experimental flow of data envelopment method.

**Figure 6:** Classification of input and output indicators.

**Figure 7:** Implementation of agricultural financial subsidy model.

**Figure 8:** Evaluation index of agricultural financial subsidy model.

**Table 1:** Hierarchy total sorting.

*W*	*B*1	*B*2	*B*3	*B*4	Weight ranking
*A*11	0.195	0	0	0	*A*23
*A*12	0.074	0	0	0	*C*11
*A*13	0.043	0	0	0	*C*32
*A*21	0	0.051	0	0	*C*31
*A*22	0	0.030	0	0	*C*12
*A*23	0	0.214	0	0	*C*21
*A*31	0	0	0.146	0	*C*13
*A*32	0	0	0.155	0	*C*22
*A*33	0	0	0.028	0	*C*33
*A*41	0	0	0	0.026	*C*41
*A*42	0	0	0	0.021	*C*42
*A*43	0	0	0	0.017	*C*43

**Table 2:** Setting of decision-making unit.

	Invest	Output		
	Amount of financial subsidy	Regional per capita income	Economic development density	Economic development depth
Income-based subsidy	12602.32	282.54	68.44	0.55
Cost-based subsidy	7242.83	127.92	63.22	0.30
Technology-based progress subsidy	9343.28	35.55	25.33	0.19
Price-based subsidy	2794.05	25.97	72.82	0.24

**Table 3:** Calculation results of relative efficiency.

	Input weight vector	Output weight vector			Relative efficiency
	Amount of financial subsidy	Regional per capita income	Economic development density	Economic development depth	
Income-based subsidy	60.89	0.0034	0	0	0.9832
Cost-based subsidy	135.45	0.0075	0	0	0.9583
Technology-based progress subsidy	79.42	0.2190	0	0	0.9023
Price-based subsidy	46.05	0	0.0218	0	0.9345

## Data Availability

The dataset can be accessed upon request.

## References

[1] Wang Y., Zhou S., Gao T. (2017). Analysis and empirical test of the influence effect of China’s agricultural subsidy policy. *Journal of Social Sciences of Jilin University*.

[2] Wang Y., Cai Y., Zhu L. (2017). Analysis of regional effects and influencing factors of agricultural subsidy policy —— taking typical main functional areas such as jingmen huanggang in wuhan, hubei Province as an example. *Journal of Huazhong Agricultural University (Social Science Edition)*.

[3] poop Ji (2006). Developing agricultural insurance to provide support for farmers’ income to grow steadily. *Journal of Dongbei University of Finance and Economics*.

[4] Wang Y., Ge J. (2009). Economic analysis of low efficiency of China’s grain subsidy policy. *Guizhou Social Sciences*.

[5] Zhang T., Guo Y., Yang J. (2018). Retrospect and prospect of China’s agricultural support and protection policy reform for 40 years (part two). *Rural Work Newsletter*.

[6] Maoqing W. (2013). *Research on the Implementation Effect of Comprehensive Subsidy Policy for Agricultural Materials in Fujian Province*.

[7] Sharma S. K. (2014). Counter-cyclical payments under doha negotiations: an analysis of agricultural subsidy programme of the US. *Agricultural Economics Research Review*.

[8] Haifa F. (2015). Thoughts and measures of agricultural subsidy system reform. *Agricultural Economic Issues*.

[9] McCloud N., Kumbhakar S. (2008). Do subsidies drive productivity? A cross-country analysis of Nordic Dairy Farms. *Bayesian Econometrics*.

[10] Yang J., Huang Z., Zhang X., Reardon T. (2013). The rapid rise of cross‐regional agricultural mechanization services in China. *American Journal of Agricultural Economics*.

[11] Zhou B. (2016). *Research Progress and Direction of Agricultural Support Policy*.

[12] Wang W. (2011). *Thoughts on China’s Agricultural Subsidy Policy under the New Situation*.

[13] Chang W. (2018). Research on regional differential financial subsidies of agricultural insurance in China. *Agricultural Economics*.

[14] Wang J., Zhou M., Wang X. (2019). Discussion on the nature and system construction of rural revitalization planning [J/OL]. *Progress of geographical science*.

[15] Ma A., Zhang A. (2012). Effect evaluation and optimization of agricultural subsidy policy. *Journal of Huazhong Agricultural University: Social Science Edition*.

[16] Yang L., Yuan X., Deng L. (2013). Efficiency evaluation of local agricultural subsidies in China based on DEA model. *Local Finance Research*.

[17] Huang D., Li X., Cai S. (2010). Research on the impact of agricultural subsidy policy on food security based on Chinese agricultural CGE model. *[J]. chinese agricultural science bulletin*.

[18] William H., Ma X. (2018). The state-of-the-art integrations and applications of the analytic hierarchy process[J]. *European Journal of Operational Research*.

[19] Jin Z., Li D., Jin Y., Ni X. (2009). The performance evaluation index and its weight calculation of local scientific research institutions —— a comparative study based on expert analysis and analytic hierarchy process. *Research on Science and Technology Management*.

[20] Pan W., Fu Q., Yang L. Research on the indicators system optimization of China national professional standardization technical committees evaluation based on AHP method.

[21] Zhang Y., Zhang R. (2021). Analysis of financial subsidy efficiency of Jilin agricultural insurance based on DEA model [J]. *Agricultural Outlook*.

[22] Qian Z., Zhang Y., Gao D. (2014). Evaluation of financial subsidy efficiency of policy-based agricultural insurance based on three-stage DEA model. *Business Research*.

